The article "Pancreatic mucinous adenocarcinoma has different clinical characteristics and better prognosis compared to non-specific PDAC: A retrospective observational study" was retracted in 2025. Reasons: unreliable results or conclusions; concerns about the authorship.

# Pancreatic mucinous adenocarcinoma has different clinical characteristics and better prognosis compared to non-specific PDAC: A retrospective observational study

**DOI:** 10.1016/j.heliyon.2024.e30268

**Published:** 2024-04-26

**Authors:** Juan Liu, Yong-jing Zhang, Jie Zhou, Zi-jian Zhang, Yu Wen

**Affiliations:** a Clinical Nursing Teaching and Research Section, Second Xiangya Hospital, Central South University, Hunan, China; b Department of Obstetrics and Gynecology, Second Xiangya Hospital, Central South University, Changsha, Hunan, China; c Department of Breast and Thyroid Surgery, Yiyang Central Hospital, Yiyang, China

**Keywords:** Pancreatic mucinous adenocarcinoma, Pancreatic ductal adenocarcinoma, Prognosis, Prognostic factors, Prediction model

## Abstract

**Background:**

Pancreatic mucinous adenocarcinoma (PMAC) is a rare malignant tumour, and there is limited understanding of its epidemiology and prognosis. Initially, PMAC was considered a metastatic manifestation of other cancers; however, instances of non-metastatic PMAC have been documented through monitoring, epidemiological studies, and data from the Surveillance, Epidemiology, and End Results (SEER) database. Therefore, it is crucial to investigate the epidemiological characteristics of PMAC and discern the prognostic differences between PMAC and the more prevalent pancreatic ductal adenocarcinoma (PDAC).

**Methods:**

The study used data from the SEER database from 2000 to 2018 to identify patients diagnosed with PMAC or PDAC. To ensure comparable demographic characteristics between PDAC and PMAC, propensity score matching was employed. Kaplan–Meier analysis was used to analyse overall survival (OS) and cancer-specific survival (CSS). Univariate and multivariate Cox regression analyses were used to determine independent risk factors influencing OS and CSS. Additionally, the construction and validation of risk-scoring models for OS and CSS were achieved through the least absolute shrinkage and selection operator-Cox regression technique.

**Results:**

The SEER database included 84,857 patients with PDAC and 3345 patients with PMAC. Notably, significant distinctions were observed in the distribution of tumour sites, diagnosis time, use of radiotherapy and chemotherapy, tumour size, grading, and staging between the two groups. The prognosis exhibited notable improvement among married individuals, those receiving acceptable chemotherapy, and those with focal PMAC (*p* < 0.05). Conversely, patients with elevated log odds of positive lymph node scores or higher pathological grades in the pancreatic tail exhibited a more unfavourable prognosis (*p* < 0.05). The risk-scoring models for OS or CSS based on prognostic factors indicated a significantly lower prognosis for high-risk patients compared to their low-risk counterparts (area under the curve OS: 0.81–0.82, CSS: 0.80–0.82).

The article "Pancreatic mucinous adenocarcinoma has different clinical characteristics and better prognosis compared to non-specific PDAC: A retrospective observational study" was retracted in 2025. Reasons: unreliable results or conclusions; concerns about the authorship.

**Conclusion:**

PMAC exhibits distinct clinical characteristics compared to non-specific PDAC. Leveraging these features and pathological classifications allows for accurate prognostication of PMAC or PDAC.

## 1 Introduction

Pancreatic cancer is reported to be the seventh leading cause of cancer-related deaths around the globe, displaying the highest fatality-to-incidence ratio among malignant tumours, with a meagre 5-year survival rate ranging from 9 % to 11 %. This condition poses a significant threat to human life and health [1,2]. Recent data indicates that China is anticipated to witness 134,374 new cases of pancreatic cancer resulting in 131,203 deaths [3], while the United States of America are expected to experience a growth in number of cases up to 62,200 and 48,800 deaths in 2023 [1,2,4]. Anticipating a steady improvement in living standards and the advent of an ageing population, it can be inferred that the risk of incidence and high mortality rates of pancreatic cancer will continue to escalate, posing a major threat to human health [5].

Indeed, the pathological classification of pancreatic cancer is highly complex, featuring remarkably heterogeneous subtypes and significant variations in prognosis. Therefore, it is imperative to investigate and summarise the epidemiological characteristics and prognostic models specific to various subtypes of pancreatic cancer. Pancreatic mucinous adenocarcinoma (PMAC), also referred to as pancreatic colloid carcinoma, represents a subtype of pancreatic ductal carcinoma originating from the pancreatic duct system [6]. Typically, it manifests in the pancreatic head, characterised by the abundant production of mucus [7]. Microscopically, PMAC is characterised by the presence of substantial mucinous pools within the tumour tissue, wherein tumour cells are either suspended or scattered along the pool periphery. On occasion, signet ring cells might also be observed [8]. Although the exact aetiology of PMAC remains unclear, being categorised under pancreatic ductal adenocarcinoma (PDAC), risk factors such as smoking [9], a high-fat diet [10], and familial inheritance [11] associated with PDAC have yet not been reported in relation to PMAC. Currently, the primary treatment approach involves a combination of modalities including surgery, chemotherapy, and radiotherapy [12,13].

However, most patients with PMAC present with extensive lesions at the initial diagnosis, and the lack of a universally accepted pathological diagnosis for PMAC contributes to the absence of a standardised management protocol. In fact, irrespective of the subtype, the prognosis for pancreatic cancer is poor; however, subtle differences in prognostic outcomes exist among different tumour subtypes. For instance, a previous study revealed that the prognosis of pancreatic signet ring cell carcinoma is worse than that of PDAC, with correlations identified through Cox model analysis involving factors such as chemotherapy and tumour size [14]. The scarcity of a standardised pathological diagnosis for PMAC renders large-scale prospective studies extremely challenging, resulting in a paucity of literature reports on PMAC. Therefore, a meticulous assessment of factors influencing prognosis becomes crucial, and the analysis of prognosis-related factors in PMAC remains an understudied domain within the unique realm of pancreatic cancer subtypes. This study aims to retrospectively analyse and determine the clinical and pathological characteristics, treatment strategies, and prognosis of patients with PMAC by comparing data from the Surveillance, Epidemiology, and End Results (SEER) database with non-specific PDAC data.

The article "Pancreatic mucinous adenocarcinoma has different clinical characteristics and better prognosis compared to non-specific PDAC: A retrospective observational study" was retracted in 2025. Reasons: unreliable results or conclusions; concerns about the authorship.

## 2 Methods and materials

### 2.1 Data source and case selection

In our study, we obtained Patient data for PMAC and PDAC from the SEER database, which is provided by the National Cancer Institute and is available on website (http://www.seer.cancer.gov). We accessed the dataset, released in November 2021 and used SEER*Stat software (v8.4.0.1) for this purpose [15]. The Medical Ethics Committee of Central South University found ethical approval for this study unnecessary because the data in the SEER database is de-identified and made openly available for public use.

Between 2000 and 2018, pancreatic cancer cases within the SEER database were identified using specific International Classification of Diseases for Oncology, third edition (ICD-*O*-3) codes: head of pancreas, body of pancreas, tail of pancreas, and pancreatic duct. Although SEER's definition of pancreatic cancer might encompass codes “islets of Langerhans” and “other specified parts of pancreas”, which capture data regarding the site of pancreatic cancer occurrence, these codes are relatively ambiguous and were not analysed in this study. The ICD-*O*-3 diagnostic codes for PMAC were mucinous adenocarcinoma and mucin-producing adenocarcinoma. For non-specific PDAC, the codes used were adenocarcinoma, not otherwise specified (NOS) and infiltrating duct carcinoma, NOS. It is worth noting that while mucinous adenocarcinoma, endocervical type is classified as mucinous adenocarcinoma, the singular sample belonging to this subtype was excluded due to its origin from the cervix. Overall survival (OS) is defined as days elapsed from the day of first diagnosis to the day of death from any cause. And cancer specific survival (CSS) is defined as days elapsed from the day of diagnosis to the day of death from pancreatic cancer [16]. Additionally, to explore the prognostic relationship between PMAC and PDAC, samples lacking OS or case-specific survival (CSS) information were excluded (Fig. 1).

The article "Pancreatic mucinous adenocarcinoma has different clinical characteristics and better prognosis compared to non-specific PDAC: A retrospective observational study" was retracted in 2025. Reasons: unreliable results or conclusions; concerns about the authorship.

**Fig. 1:** The mind map of this study. C250: head of pancreas; C251: body of pancreas; C252: tail of pancreas; C253: pancreatic duct; 8140/3: adenocarcinoma, not otherwise specified (NOS); 8500/3: infiltrating duct carcinoma, NOS; 8480/3: mucinous adenocarcinoma; 8481/3: mucin-producing adenocarcinoma; 8482/3: mucinous adenocarcinoma, endocervical type; PSM: propensity score matching; KM analysis: Kaplan-Meier analysis; LASSO: least absolute shrinkage and selection operator regression.

### 2.2 Clinical information collection and processing

In our study, we obtained the following variables from SEER database: firstly, we obtained demographic information which included patient identity, gender, the year of diagnosis, age of patient at diagnosis, financial status, general characteristics of the tumour which included (histological type, primary site of tumour, size, number of tumours, grade, tumour-node-metastasis [TNM] staging, summary staging, sequence number, lymph node ratio [LNR], and log odds of positive lymph node [LODDS]), basic information about the type of treatment received such as (radiation and chemotherapy), and the recorded data of survival based of follow-up which included (overall survival and cause-specific survival). Additionally, we calculated LNR and LODDS using the number of lymph nodes and positive lymph nodes detected based on the data collected from the SEER database, which contributed to the establishment of a novel lymph node metastasis staging system [17]. LNR represents the ratio of histopathological positive lymph nodes to total retrieved lymph nodes, while LODDS is calculated by formula as log [(positive lymph nodes + 0.5)/(negative lymph nodes + 0.5)]. As the effectiveness of LNR and LODDS is already established knowledge as prognostic factors across various malignancies [17,18], this study further investigated their applicability in predicting the prognosis of PDAC and PMAC specifically.

In the next phase after data acquisition, the variables were categorised for subsequent analysis. Additionally, we used X-tile software (v3.6.1) to determine the optimal cut-off values for continuous variables such as (year of diagnosis, age at diagnosis, tumour size, LNR, and LODDS) based on different survival times. Continuous variables were then converted into categorical variables using the optimal cut-off values. For instance, “year of diagnosis” was divided into "≤2004″, "2004–2010″, and ">2010"; age at diagnosis (years) was divided into "≤68″, "68–81″, and ">81"; tumour size (mm) was divided into "≤20″, "20–85″, ">85″, and "unknown"; LNR was divided into "≤0.2″, "0.2–0.8″, ">0.8″, and "unknown"; and LODDS was divided into "≤-1.0″, "-1.0–0.5″, ">-0.5″, and “unknown” (Fig. 2A–E).

The article "Pancreatic mucinous adenocarcinoma has different clinical characteristics and better prognosis compared to non-specific PDAC: A retrospective observational study" was retracted in 2025. Reasons: unreliable results or conclusions; concerns about the authorship.

**Fig. 2:** Determining of the optimum cut-off values for the variables. (A) Kaplan–Meier (KM) analysis of pancreatic mucinous adenocarcinoma patient distribution according to age via X-tile software analysis. (B) KM analysis of patient distribution according to the lymph node ratio (LNR). (C) KM analysis of patient distribution according to the log odds of positive lymph node (LODDS). (D) KM analysis of patient distribution according to the tumour size. (E) KM analysis of patient distribution according to the diagnostic years. pval: *p* value; HR: hazard ratio; CI: confidence interval.

### 2.3 Propensity score matching (PSM) and survival analysis

To comprehensively investigate the prognostic factors associated with PMAC, our objective was to incorporate a broad spectrum of patient characteristics. Due to potential heterogeneity in the baseline characteristics of patients with PDAC and PMAC, it is necessary to balance and screen patient information based on the baseline data using PSM analysis. The PSM approach involves constructing a binary logit model with survival time as the dependent variable (Y) and other factors as independent variables (X). The model generates a predicted value, known as the PSscore value. Matching is considered successful when the PSscore falls within an acceptable calliper value. Changes before and after matching are then compared, and the matching effect is assessed using the *p*-value and standardised mean difference (SMD) value [19]. It was found that excluding patient information with missing household income was crucial to ensure the presence of information for each subgroup of feature values after PSM. Therefore, in this step, samples without household income data were initially excluded (8480/3: n = 1; 8140/3: n = 5).

The R package “MatchIt” (v4.1.0) was used to perform PSM with a 1:1 matching ratio and a calliper of 0.05 for all the aforementioned variables [19]. In the results, if the *p*-value was less than 0.05 or the SMD was less than 0.1 in the results, it was considered that there was no difference in the sample features. Conversely, if either condition was not met, it was deemed that there was a difference in the sample features [20]. For this study, the endpoints were set as OS and CSS. Survival curves were constructed using the Kaplan–Meier (KM) analysis, and a gehan-breslow or log-rank test was employed to compare patients with PMAC and PDAC.

The article "Pancreatic mucinous adenocarcinoma has different clinical characteristics and better prognosis compared to non-specific PDAC: A retrospective observational study" was retracted in 2025. Reasons: unreliable results or conclusions; concerns about the authorship.

### 2.4 Univariate and multivariate cox regression analysis

After comparing the survival differences between patients with PDAC and PMAC before and after PSM, an additional step involved delving into potential clinical features influencing PMAC survival. Initially, univariate Cox regression analysis was employed to investigate the corelation between all clinical features and prognosis in patients with PMAC, with potential prognostic factors (*p* < 0.05) undergoing preliminary screening. In univariate Cox analysis, a feature variable is considered prognostically relevant if it satisfies *p* < 0.05 and the confidence interval (CI) of the hazard ratio (HR) is both greater than and less than 1. For multiple categorical feature variables, if one group meets the aforementioned conditions, all groups of that variable are included in subsequent multivariate Cox analysis. Subsequently, significant features identified in the univariate Cox regression analysis were incorporated into the multivariate Cox regression analysis to determine the independent risk factors for all PMAC cases [21].

### 2.5 Least absolute shrinkage and selection operator (LASSO) regression analysis and construction of a nomogram

Based on the earlier mentioned multivariate Cox regression analysis, a simple prognostic prediction system for PMAC could be constructed. However, recognising the potential collinearity interference in multivariate Cox regression analysis and the survival differences between PMAC and PDAC, it was believed that a more comprehensive prediction model could be established by integrating the data from PSM-adjusted PMAC and PDAC. The LASSO regression, an algorithm integrating an L1 regularisation term into the ordinary least squares method, was deemed suitable for this process. LASSO regression is a shrinkage algorithm to achieve feature selection in the Cox model [22,23]. This allows certain feature variables’ coefficients to be compressed to zero, facilitating the automatic selection of feature variables.

After PSM and uni/multi-variate Cox regression analysis, LASSO regression analysis was used to find out the optimal weighted coefficients for different pathological types of pancreatic cancers and their clinical features. A model was then established to determine whether these features could specifically predict the prognosis of patients with PMAC and PDAC. Using the R package “glmnet”, the LASSO regression model for OS and CSS of patients with PMAC and PDAC was established using 10X cross-validation [24]. It is noteworthy that for multi-class non-ordinal variables, a covariate matrix transformation was required before inclusion in the LASSO analysis. In the analysis outcomes, if any variable within the covariate matrix was included in the LASSO model, the entire variable needed to be included in the final modelling. Furthermore, the optimal λ values were defined as 0.0033 and 0.0030 for OS and CSS, respectively.

The article "Pancreatic mucinous adenocarcinoma has different clinical characteristics and better prognosis compared to non-specific PDAC: A retrospective observational study" was retracted in 2025. Reasons: unreliable results or conclusions; concerns about the authorship.

Subsequently, the receiver operating characteristic (ROC) curve for the risk score model was analysed using the R package "pROC", and the area under the curve (AUC) and its corresponding CI were determined. Patients were divided into two groups (high- and low-risk) based on the optimal cut-off value or the median of the risk score. Based on the R package "survival", further analysis of KM survival differences between the two groups was conducted. Lastly, R package “rms” was used to integrated the prognostic data and perform a nomogram, which calculates disease risk or individual survival probability.

## 3 Results

### 3.1 Comparison of baseline clinical characteristics between PMAC and PDAC

This study included 88,202 patients (3345 patients with PMAC and 84,857 patients with PDAC) from the SEER database (Fig. 1). Significant differences were observed in 15 baseline clinical characteristics between the PDAC and PMAC groups (*p* < 0.05; Fig. 2A–E, Fig. 3, Supplementary Table 1). For example, the proportion of PDAC cases occurring in the pancreatic head was significantly higher than that of PMAC cases (67.0 % vs. 60.7 %, *p* < 0.001). Over the period from 2000 to 2018, the number and proportion of PDAC diagnoses increased, while the proportion of PMAC diagnoses exhibited no significant change. Furthermore, the PMAC group showed a lower proportion of patients receiving radiation or chemotherapy compared to the PMAC group (*p* < 0.001). In terms of tumour characteristics, the proportion of patients with PDAC with tumour sizes ranging from 20 to 85 mm was higher than that of patients with PMAC (75.3 % vs. 66.8 %, *p* < 0.001). Additionally, the proportion of patients with Grade I PDAC was lower than that of patients with PMAC (3.7 % vs. 9.3 %). Significant differences in TNM staging were observed between the two groups (*p* < 0.005), with lower proportions of T0/Ti/TX, N0, and M0 in the PMAC group compared to the PDAC group. Interestingly, PMAC exhibited a higher proportion of distant metastases (56 % vs. 43.6 %), and the proportion of localised tumours was significantly lower in PMAC than in PDAC (28.4 % vs. 32.9 %). However, certain variables, including surgical treatment, race, marital status, median household income, and sex distribution, demonstrated similarities between the two groups.

The article "Pancreatic mucinous adenocarcinoma has different clinical characteristics and better prognosis compared to non-specific PDAC: A retrospective observational study" was retracted in 2025. Reasons: unreliable results or conclusions; concerns about the authorship.

**Fig. 3:** Consistency of pancreatic mucinous adenocarcinoma and pancreatic ductal adenocarcinoma feature distribution before and after propensity score matching. Standardised mean difference>0.1 indicates heterogeneity in the sample distribution, while conversely, it is considered balanced in the sample distribution. M: metastasis stage; T: tumor stage; N: lymph node staging; Surg.Rad: surgery or radiation.

### 3.2 PSM and survival analysis

Firstly, use PSM to balance the clinical baseline characteristics of the two types of tumours (all standard deviations <0.05; Fig. 3, Supplementary Table 1). Subsequently, 6674 patients (3337 with PMAC and 3337 with PDAC) were included after PSM analysis. KM survival analysis was performed on patients with PMAC and PDAC after PSM. Before PSM, the analysis included 88,202 patients, revealing median OS and CSS durations of 6 months for both the PMAC and PDAC groups. The PMAC group with 1-year, 3-year, and 5-year OS rates of 31.97 %, 11.62 %, and 8.02 % exhibited a slightly better prognosis compared to PDAC (*p* = 0.011). Similarly, 1-year and 3-year CSS rates were 36.26 % vs. 33.59 %, 14.50 % vs. 10.11 %, and 10.84 % vs. 6.47 %, respectively (*p* = 0.0027; Fig. 4A and B).

**Fig. 4:** Survival differences between pancreatic mucinous adenocarcinoma (PMAC) and pancreatic ductal adenocarcinoma (PDAC) patients before and after propensity score matching (PSM). Overall survival (OS) (A) and cancer-specific survival (CSS) (B) of patients with PMAC and PDAC before PSM. OS (C) and CSS (D) of patients with PMAC and PDAC after PSM. Gehan–Breslow tests were used to generate the *p*-values.

In the PSM-adjusted cohort of 6674 patients, despite similar median OS and CSS times, the PMAC group exhibited a slightly superior prognosis at 1, 3, and 5 years. After PSM, the median OS and CSS were 6 months and 7 months for the PMAC and PDAC groups, respectively. Moreover, the 1-year, 3-year, and 5-year OS rates were 31.96 % vs. 28.25 %, 11.62 % vs. 8.00 %, and 8.01 % vs. 4.65 % for the PMAC and PDAC groups, respectively (*p* < 0.0001). The 1-year and 3-year CSS rates were 36.20 % vs. 31.76 %, 14.48 % vs. 10.08 %, and 10.81 % vs. 6.31 %, respectively (*p* < 0.0001; Fig. 4C and D). These findings indicate that the prognosis of PDAC patients was slightly less favourable than that of patients with PMAC before and after PSM. However, after mitigating the effects of demographic information, tumour characteristics, and treatment information through PSM, this difference in prognosis became more significant, further confirming that PMAC exhibits a more favourable prognosis compared to the common PDAC pathological type.

The article "Pancreatic mucinous adenocarcinoma has different clinical characteristics and better prognosis compared to non-specific PDAC: A retrospective observational study" was retracted in 2025. Reasons: unreliable results or conclusions; concerns about the authorship.

### 3.3 Univariate and multivariate analysis

Subsequently, separate univariate and multivariate Cox regression analyses were conducted for OS and CSS to identify potential clinical features influencing the prognosis of patients with PMAC. The univariate regression analysis for OS and CSS revealed that year of diagnosis, primary site, LNR, LODDS, surgery with radiation, radiation, chemotherapy, tumour size, sequence number, total number of tumours, race, marital status, median household income, age, grade, summary stage, TNM stage, and sex were prognostic factors for patients with PMAC (Fig. 5, Supplementary Table 2). A later diagnosis time, undergoing surgery, radiation and chemotherapy, having multiple tumours, and presenting with localised tumours were identified as potential protective factors for PMAC prognosis, whereas high LNR, elevated LODDS, larger tumour size, older age, higher pathological grade, and advanced N/M stage were all potential risk factors for prognosis (*p* < 0.05).

**Fig. 5:** Forest map of the univariate Cox regression analysis for PMAC. Only feature information with *p* < 0.05 is presented. DSW: divorce/separation/widow.

In the multivariate regression analysis for overall survival (OS), several factors were assessed in comparison to the reference index. The results indicated that the diagnosis year after 2010 (HR = 0.84, 95 % CI: 0.73–0.98), and like most of the other tumours,receiving chemotherapy (HR = 0.52, 95 % CI: 0.48–0.56), having multiple primary tumours (HR = 0.33, 95 % CI: 0.15–0.74), presenting with localized tumours (HR = 0.42, 95 % CI: 0.35–0.52), and regional tumours (HR = 0.70, 95 % CI: 0.62–0.80) were identified as independent protective factors for prognosis and significantly contributed to better prognosis. It is noteworthy that marietal status (being married, HR = 0.85, 95 % CI: 0.78–0.93) was unusually identified as independent protective factors and helped in better prognosis. It is also noteworthy that T3 was not considered a protective factor compared to T0/Ti/TX due to the complexity and potential bias associated with the T0/Ti/TX components.

Conversely, certain factors were identified as independent risk factors for prognosis compared to the reference index. These include the usual tumor characteristics such as location i.e. tumours in the pancreatic tail (HR = 1.21, 95 % CI: 1.11–1.33), lymph node involvement i.e. lymph node ratio (LODDS) between −1.0 and −0.5 (HR = 1.71, 95 % CI: 1.37–2.14), LODDS greater than −0.5 (HR = 2.33, 95 % CI: 1.70–3.20) with higher lymph node involvement contributing to poorer prognosis, tumor grading i.e. grade 2 (HR = 1.23, 95 % CI: 1.06–1.43), grade 3 (HR = 1.48, 95 % CI: 1.26–1.75) with higher grading contributing to higher risk and poorer prognosis, and tumor staging i.e. M1 stage (HR = 1.21, 95 % CI: 1.05–1.38) with more advanced stage resulting in poorer prognosis. Like most of the other tumours, age between 68 and 81 years (HR = 1.31, 95 % CI: 1.20–1.44) was also identified as independent risk factor for prognosis compared to the reference index where elder age was related to poorer prognosis. For more detailed information, refer to Fig. 6 and Supplementary Table 3 in the manuscript.

The article "Pancreatic mucinous adenocarcinoma has different clinical characteristics and better prognosis compared to non-specific PDAC: A retrospective observational study" was retracted in 2025. Reasons: unreliable results or conclusions; concerns about the authorship.

**Fig. 6:** Forest map of multivariate COX regression analysis for pancreatic mucinous adenocarcinoma. Only feature information with *p* < 0.05 is presented.

In the multivariate regression analysis for cancer-specific survival (CSS), various factors were evaluated in comparison to the reference index. The findings revealed that several factors were independent protective factors for prognosis. These included the diagnosis year after 2010 (HR = 0.82, 95 % CI: 0.70–0.96). Like general trend in oncology, some factors such as receiving chemotherapy (HR = 0.53, 95 % CI: 0.48–0.57), having multiple primary tumours (HR = 0.40, 95 % CI: 0.18–0.90), presenting with localized tumours (HR = 0.41, 95 % CI: 0.33–0.51), and regional tumours (HR = 0.69, 95 % CI: 0.60–0.79) were identified as independent protective factors for prognosis. Here also, being married (HR = 0.89, 95 % CI: 0.81–0.98) was unusually identified as independent protective factors and helped in better prognosis. Remarkably, these protective factors were consistent with the results of the overall survival (OS) analysis. Similarly, T1 and T3 stages were not considered protective factors for CCS compared to T0/Ti/TX, despite their statistically significant values.

Conversely, certain factors were identified as independent risk factors for prognosis compared to the reference index. These include the tumor characteristics such as tumor location i.e. tumours in the pancreatic tail (HR = 1.20, 95 % CI: 1.09–1.33), lymph node invovement i.e. lymph node ratio (LODDS) between −1.0 and −0.5 (HR = 1.82, 95 % CI: 1.42–2.33), LODDS greater than −0.5 (HR = 2.62, 95 % CI: 1.82–3.68), where higher lymph node involvement was related to poorer prognosis, grade 2 (HR = 1.25, 95 % CI: 1.07–1.48), grade 3 (HR = 1.51, 95 % CI: 1.27–1.80), grade 4 (HR = 1.82, 95 % CI: 1.05–3.13) where higher tumor grade was related to poorer prognsis, and M1 stage (HR = 1.21, 95 % CI: 1.04–1.40) where advaned tumor stage was related to poorer prognosis. Here also, age was also identified as an independent risk factor for prognosis i.e. between 68 and 81 years (HR = 1.26, 95 % CI: 1.14–1.39) indicating elder age was related to poorer prognosis. Notably, grade 4 emerged as a unique independent risk factor for CCS prognosis, while all other risk factors were consistent with those for OS (see Fig. 6 and Supplementary Table 3 for detailed information).

The article "Pancreatic mucinous adenocarcinoma has different clinical characteristics and better prognosis compared to non-specific PDAC: A retrospective observational study" was retracted in 2025. Reasons: unreliable results or conclusions; concerns about the authorship.

### 3.4 Construction of PDAC and PMAC operating systems and CSS prediction models

Using the prognostic factors identified through univariate analysis, LASSO regression analysis was conducted to develop predictive models for OS and CSS models that simultaneously encompass PDAC and PMAC. The OS prediction model (Fig. 7A and B) and CSS model (Fig. 8A and B) were performed by assimilating crucial prognostic factors and pathological grouping data. After ten-fold cross-validation, the optimum λ values for the OS and CSS models were 0.0033 and 0.0030, respectively. Finally, 20 prognostic factors were included in the prediction model of OS, encompassing group, year of diagnosis, age, grade, summary stage, TNM stage, and so on.

**Fig. 7:** Constructing and evaluating OS predictive models in datasets after PSM. (A, B) The coefficient and deviance profile of LASSO analysis. (C) KM analysis revealing the differences of OS between the low-(L) and high-(H)score calculated by the LASSO model. (D) ROC of OS at 1to 9-years according to the risk score in the LASSO model. LASSO: least absolute shrinkage and selection operator; AUC: area under the curve; ROC: Receiver operating characteristic curves.

**Fig. 8:** Constructing and evaluating CSS predictive models in datasets after PSM. (A, B) The coefficient and deviance profiles of LASSO analysis. (C) KM analysis revealing the differences of OS between the low-(L) and high-(H)score calculated by the LASSO model. (D) ROC of CSS at 1 to 9-years according to the risk score in the LASSO model.

Furthermore, survival analysis based on risk scores was conducted on 6674 patients screened by PSM. The optimal threshold value for the OS model was determined to be −0.1629. Patients were then categorised into high-risk and low-risk groups based on the optimal threshold value. KM curve analysis demonstrated that the OS model effectively distinguished between patients with favourable and unfavourable prognosis, with the low-risk group exhibiting longer OS compared to the high-risk group (HR = 3.39, 95 % CI: 2.37–4.85, *p* = 2.4e-12; Fig. 7C). Similarly, based on the median risk score, patients with high- or low-score were conducted to survival analysis. And results revealed that the OS of the low-score group was longer than the other (HR = 3.09, 95 % CI: 2.30–4.15, *p* = 5.1e-15). Time-dependent ROC analysis illustrated that the AUC values for the 1 to 9-year OS risk scores were 0.81–0.82 (Fig. 7D).

The article "Pancreatic mucinous adenocarcinoma has different clinical characteristics and better prognosis compared to non-specific PDAC: A retrospective observational study" was retracted in 2025. Reasons: unreliable results or conclusions; concerns about the authorship.

Similarly, the CSS prediction model identified 20 prognostic factors (Fig. 8A and B). These 20 factors identified by the OS prediction model were also included in the CSS prediction model. Based on the optimal threshold value (15.2866) (HR = 3.75, 95 % CI: 3.51–4.01, *p* < 0.0001) or median risk score (HR = 3.13, 95 % CI: 2.96–3.31, *p* < 0.0001), the high-risk group exhibited a shorter CSS compared to the low-risk group (Fig. 8C), b. For the CSS prediction model, the AUC values for the 1-, 3-, 5-, 7-, and 9-year CSS risk scores were 0.80, 0.82, 0.82, 0.82, and 0.82, respectively (Fig. 8D).

### 3.5 Validation and visualisation of OS and CSS prediction models

In our study, the LASSO-Cox results were presented using nomograms to improve the practicality of the aforementioned models, and calibration curves were used to demonstrate the effectiveness of the prediction models (Fig. 9). The prognostic factors for OS and CSS were identified via LASSO regression analysis, followed by additional Cox analysis on the selected factors in OS and CSS. The R package “rms” was used to integrate survival information, and feature scores, leading to the establishment of OS and CSS column charts along with corresponding calibration curves. The results from the column charts indicated that by calculating the total score based on specific patient features and determining the corresponding survival rate, the 1-, 3-, and 5-year OS or CSS rates of patients with PDAC and PMAC can be quickly and easily predicted (Fig. 9). The overall C-index for the OS and CSS predictive models were 0.7539 (95 % CI: 0.7473–0.7606, *p* < 0.0001) and 0.7545 (95 % CI: 0.7475–0.7615, *p* < 0.0001), respectively (Fig. 9).

**Fig. 9:** The universal nomogram predicting PMAC and PDAC based on survival-associated predictive models.

## 4 Discussion

Ductal adenocarcinoma stands as the predominant malignant tumour within the exocrine pancreas, with other less prevalent histological subtypes encompassing mucinous cystadenocarcinoma, colloid carcinoma, intraductal papillary mucinous carcinoma, acinar cell carcinoma, and other rare subtypes [25]. According to the World Health Organisation International Histological Classification, colloid carcinoma also referred to as PMAC, is categorised under the PDAC subtype [6,26]. Similarly, in the SEER database classification, mucinous adenocarcinoma is a special subtype different from pancreatic non-specific adenocarcinoma or intraductal carcinoma. Despite having a higher incidence in the SEER database compared to mucinous cystadenocarcinoma or intraductal papillary mucinous carcinoma, mucinous adenocarcinoma is rarely discussed in clinical contexts and is often confused with PDAC. However, our study revealed divergent prognosis between patients with PMAC and PDAC before and after PSM matching, underscoring the need for increased attention to this subtype by clinicians. Currently, the comprehension of these tumours primarily relies on limited single-institution case reports, with mucinous adenocarcinoma being less frequently addressed in epidemiological studies compared to mucinous cystadenocarcinoma and intraductal papillary mucinous carcinoma. Given the rarity of this tumour, the objective of this population-based retrospective study is to investigate the relationship between the clinical and pathological characteristics and the survival rate of patients with PMAC.

The article "Pancreatic mucinous adenocarcinoma has different clinical characteristics and better prognosis compared to non-specific PDAC: A retrospective observational study" was retracted in 2025. Reasons: unreliable results or conclusions; concerns about the authorship.

Among all prognostic features, paramount considerations include tumour size, lymph nodes, and metastasis. Specifically, the prevalence of patients with PDAC with tumour sizes ranging from 20 to 85 mm surpasses that of patients with PMAC (75.3 % vs. 66.8 %, *p* < 0.001). The actual tumour size of non-specific PDAC reported in previous studies ranges from 0 to 130 mm, with an average of 25 mm. Another study corroborated average actual and computed tomography sizes for PDAC at 29 mm and 30 mm, respectively [27]. In our study, LODDS values exceeding −1.0 emerged as a prognostic risk factor, underscoring the significant impact of varying LODDS values on prognostic assessment in PMAC. The literature on LODDS in pancreatic cancer remains limited, with Dimitrios et al. [17] evaluating the relationship between LNR and LODDS and prognosis in 319 patients with PDAC, revealing statistically significant outcomes exclusively for LODDS classification. Lee et al. [28], in their examination of pancreatic cancer LODDS values categorised as < -3.5, −3.5 to −0.970, and >-0.97, reported an ROC AUC of 0.596. Our findings provide further support for the predictive utility of LODDS in the context of PMAC.

Interestingly, PMAC exhibits a higher incidence of distant metastasis (56 % vs. 43.6 %), while the proportion of localised tumours in PMAC is significantly lower than that in PDAC (28.4 % vs. 32.9 %). Although this outcome might appear inconsistent with the superior prognosis of PMAC compared to PDAC, it is crucial to consider the potential bias introduced by the fact that 16.5 % of patients with PDAC have an unknown metastasis status. Either epidemiological data indicates that 40.2 % present with localised tumours, 8.1 % exhibit regional disease, and 49.6 % manifest distant metastasis [29,30]. The result concerning distant metastasis in this study falls between the findings for PMAC and PDAC. Another finding is that patients with localised tumours (HR = 0.41, 95 % CI: 0.33–0.51) and regional tumours (HR = 0.69, 95 % CI: 0.60–0.79) experience significantly improved prognosis compared to those with distant metastasis. This observation is reflected in TNM staging, where the M1 stage (HR = 1.21, 95 % CI: 1.04–1.40) emerges as an independent prognostic risk factor for PMAC. This corroborates findings from numerous studies on PDAC [[31], [32], [33]], underscoring the limited efficacy of current treatment modalities in managing advanced PDAC.

The article "Pancreatic mucinous adenocarcinoma has different clinical characteristics and better prognosis compared to non-specific PDAC: A retrospective observational study" was retracted in 2025. Reasons: unreliable results or conclusions; concerns about the authorship.

Regarding tumour grading, after excluding patients with unknown pathological grades, patients with grade I and II PDAC constituted 57.8 %, whereas known graded PMAC patients comprised 69.8 % with grade I and II combined. Earlier publications provided a cumulative estimate of 66.1 % for PDAC [34]. It is noteworthy that tumour grading data has been rarely reported in previous case series. Additionally, pathological grading of grades II–IV emerged as a relative risk factor when compared to grade I, with age demonstrating a significant association with prognosis [35,36].

In our study, pancreatic tail tumours (HR = 1.20, 95 % CI: 1.09–1.33) were identified as a prognostic risk factor for PMAC. The literature presents conflicting findings regarding the relationship between the location of pancreatic tumours and prognosis [37]. Similar to our findings, David et al. [37] reported that head tumours exhibited a better prognosis than body/tail tumours in PDAC (2-year OS, 44 vs. 27 %, *p* = 0.043). Additionally, Zhang et al. [38] found that pancreatic body/tail cancers demonstrated significantly more enriched genomic alterations in KRAS (97.1 % vs. 82.4 %, *p* = 0.004) and mothers against decapentaplegic homolog 4 (42.0 % vs. 21.2 %, *p* = 0.008) compared to pancreatic head cancers. Furthermore, Ge et al. [39] observed markedly superior overall survival and objective response rates in patients with pancreatic body/tail cancer compared to those with pancreatic head cancer.

Beyond the fundamental attributes of tumours, treatment modalities play a crucial role in influencing the prognosis of PMAC. The rarity of these tumours, constituting only 3.9 % of all pancreatic malignancies according to the SEER database, has led to limited evaluations of treatment methods and prognoses for PMAC. In this study, the largest PMAC patient cohort was presented and its clinical and pathological characteristics and survival rates were investigated. Despite the higher occurrence of PDAC in the pancreatic head compared to PMAC (67.0 % vs. 60.7 %, *p* < 0.001), the pancreatic head remains the primary site of PMAC occurrence, aligning with previous reports [37]. Similar to numerous PDAC studies [40,41], it was observed that chemotherapy benefits patients (HR = 0.53, 95 % CI: 0.48–0.57); however, this conclusion specifically applies to PMAC. Interestingly, radiotherapy and surgical treatment did not manifest as protective factors for PMAC, potentially attributable to a preponderance of late-stage cases in the SEER database, making it challenging for these cases to derive benefit from surgery and radiotherapy. Effective surgery can significantly prolong the survival time of patients (non-surgery vs. surgery: 4 vs. 16 months) [42]. Tadashi et al. [12,13] reported a patient who underwent FOLFRINOX and subsequently underwent surgical resection of the tumour, experiencing no disease progression within 10 months after surgery. Additionally, the first of two or more primaries (HR = 0.40, 95 % CI: 0.18–0.90) emerged as a protective factor for PMAC. However, in small cell lung cancer studies, this situation appears to be a prognostic risk factor, necessitating further confirmation of its protective effect [43].

The article "Pancreatic mucinous adenocarcinoma has different clinical characteristics and better prognosis compared to non-specific PDAC: A retrospective observational study" was retracted in 2025. Reasons: unreliable results or conclusions; concerns about the authorship.

In this study, marital status (HR = 0.89, 95 % CI: 0.81–0.98) emerges as a protective factor for PMAC, aligning with previous analyses of PDAC [42]. These studies found that irrespective of whether patients with PDAC underwent surgery, married individuals exhibited a median survival time of 1–3 months longer than their unmarried counterparts. The potential benefit of marriage on pancreatic cancer prognosis might stem from emotional support within spousal and familial relationships, although no specific research has explored this aspect.

Some studies have used the above prognostic factors and other similar factors to construct a prognostic model for pancreatic cancer. For instance, Ge et al. [44], using carbohydrate antigen 19-9, vascular recovery, tumour differentiation, LNR, and advanced chemotherapy, formulated a postoperative prognosis model for PDAC with a CI value of 0.65 (equivalent to the AUC). Furthermore, studies have used SEER data to develop prognostic models for rare subtypes, such as pancreatic signet ring cell carcinoma [14]. This study used data such as LODDS, tumour size, age, and T-stage to construct a prognostic model, with an AUC value ranging between 0.79 and 0.89. Our study is the first to present a prognostic model for PMAC (AUC: 0.79–0.83). However, this study has limitations due to the lack of external data validation. Future validations should involve larger samples and more comprehensive data to verify and refine our conclusions.

In conclusion, given the variations in survival and epidemiological characteristics between PMAC and non-specific PDAC, our study confirms the need to explore the special prognostic factors associated with this subtype. Notably, our findings reveal that being married and receiving acceptable chemotherapy significantly contribute to a more favourable prognosis for patients with focal PMAC. Conversely, tumours in the pancreatic tail, elevated LODDS scores, or higher pathological grades were associated with markedly unfavourable outcomes. Therefore, early chemotherapy for localised PMAC could substantially prolong patient survival, and maintaining a stable marital status also emerges as a beneficial factor for the prognosis of patients with PMAC.

The article "Pancreatic mucinous adenocarcinoma has different clinical characteristics and better prognosis compared to non-specific PDAC: A retrospective observational study" was retracted in 2025. Reasons: unreliable results or conclusions; concerns about the authorship.

## Funding

This work was supported by 10.13039/501100004735Natural Science Foundation of Hunan Province, No. 2023JJ30789 and 2021SK52602; and 10.13039/100016802Natural Science Foundation of Changsha No. kq2208338; and Health Research Project of Hunan Provincial Health Commission, No. 20201421 and 202304017215.

## Data availability statement

The datasets generated and/or analysed during the current study are available in the Surveillance, Epidemiology, and End Results database, [https://seer.cancer.gov/].

## CRediT authorship contribution statement

**Juan Liu:** Writing – review & editing, Data curation, Conceptualization. **Yong-jing Zhang:** Resources, Funding acquisition, Data curation. **Jie Zhou:** Software, Funding acquisition, Data curation. **Zi-jian Zhang:** Writing – original draft, Methodology, Conceptualization. **Yu Wen:** Validation, Supervision, Project administration, Funding acquisition.

## Declaration of competing interest

The authors declare that they have no known competing financial interests or personal relationships that could have appeared to influence the work reported in this paper.
